# Prediction of Bronchopneumonia Inpatients' Total Hospitalization Expenses Based on BP Neural Network and Support Vector Machine Models

**DOI:** 10.1155/2022/9275801

**Published:** 2022-05-18

**Authors:** Cuiyun Wu, Dahui Zha, Hong Gao

**Affiliations:** The Third People's Hospital of Hefei, Hefei, Anhui 230022, China

## Abstract

**Objective:**

BP neural network (BPNN) model and support vector machine (SVM) model were used to predict the total hospitalization expenses of patients with bronchopneumonia.

**Methods:**

A total of 355 patients with bronchopneumonia from January 2018 to December 2020 were collected and sorted out. The data set was randomly divided into a training set (*n* = 249) and a test set (*n* = 106) according to 7 : 3. The BPNN model and SVM model were constructed to analyze the predictors of total hospitalization expenses. The effectiveness was compared between these two prediction models.

**Results:**

The top three influencing factors and their importance for predicting total hospitalization cost by the BPNN model were hospitalization days (0.477), age (0.154), and discharge department (0.083). The top 3 factors predicted by the SVM model were hospitalization days (0.215), age (0.196), and marital status (0.172). The area under the curve of these two models is 0.838 (95% CI: 0.755~0.921) and 0.889 (95% CI: 0.819~0.959), respectively.

**Conclusion:**

Both the BPNN model and SVM model can predict the total hospitalization expenses of patients with bronchopneumonia, but the prediction effect of the SVM model is better than the BPNN model.

## 1. Introduction

Bronchopneumonia (also known as lobular pneumonia) is one of the most common respiratory infections [1], with an incidence rate of more than 20% [2]. Bronchopneumonia is a severe disease that threatens people's health in China. It is also a disease that accounts for a large proportion of the spectrum of hospitalized infections [3, 4]. Bronchopneumonia is often caused by bacteria, viruses, molds, mycoplasma pneumonia, and other pathogens. It can also be “a mixed infection” by viruses and bacteria [5]. After the onset, the inflammation of lung tissue thickens the respiratory membrane and blocks the lower respiratory tract, causing dysfunction of ventilation and ventilation. The clinical manifestations are fever, cough, and shortness of breath [2].

The aging stage with the highest incidence of bronchopneumonia among children is 5 ~ 9 years old, and the onset age of patients gradually decreases [6]. Once infected, it will affect patients' quality of life and bring a certain economic burden to families. In addition, the disease can cause pressure on the national medical insurance fund [7, 8]. Therefore, strengthening the cost research of bronchopneumonia and formulating effective intervention measures can reduce the economic burden on patients and medical insurance [9].

Data mining is a process that combines artificial intelligence and database technology to extract potentially valuable information from a large number of complex and fuzzy data [10–14]. The application of artificial intelligence in the medical field is gradually maturing. BP neural network (BPNN) model [15] and support vector machine (SVM) model [16] have no special requirements for data distribution and have certain fault tolerance. In addition, they are widely used in dealing with complex relationships between data and can seek the optimal solution under the current information [17]. Thus, this study used these two models to predict the total hospitalization cost of patients with bronchopneumonia and compared the prediction efficiency of the two models.

## 2. Methods

### 2.1. General Information

A total of 355 patients with bronchopneumonia who were mainly diagnosed as discharged from the first page of medical records from a grade III class hospital in Anhui province from January 2018 to December 2020 were collected. Inclusion criteria: (1) inpatients; (2) the diagnosis was bronchopneumonia. Exclusion criteria: (1) length of stay was 1 day; (2) it costs more than 40,000 yuan.

### 2.2. Research Indicators

The preliminary included research indicators include medical payment method, hospitalization times, sex, age, nationality, occupation, marital status, admission way, admission situation, whether to change majors, discharge departments, actual hospitalization days, whether to implement clinical pathway management, whether to complete clinical pathway, whether to have complications, whether to be critically ill or seriously ill during hospitalization, whether to meet the outpatient discharge diagnosis, whether to meet the admission and discharge diagnosis, admission condition, and whether to merge. The dependent variable is the total hospitalization expenses.

### 2.3. Partition of Data Set

Since the model construction of deep learning depends on the training of a large amount of data, it has the problem of uneven data distribution. Therefore, it is necessary to preprocess the data set. To prevent overfitting, this study verified the included data by a 10-fold crossover method. That is to say, it is divided according to the ratio of 7 : 3 to form a training set and a test set [18]. Among the patients, 70% of the data sets were used for the training set (*n* = 249) and 30% for the test set (*n* = 106).

### 2.4. Construction of Prediction Model

#### 2.4.1. BP Neural Network Model

Total hospitalization expenses were used as the output variable, and statistically significant variables in univariate analysis were used as input variables. The hidden layer activation function is the hyperbolic tangent function, and the output layer activation function is the identity function. The data set is divided into the training set and test set, and the prediction model and BPNN model are constructed, respectively. The accuracy of the network will be calculated based on the verification set, where the relative error is the proportion of the sum of squares of the residuals and mean deviations to the sum of squares of the dependent variables. The prediction accuracy is 1-relative error [19]. After the network training is completed, the importance of each input variable to the prediction of the target variable is judged to reflect the relative effect of the input variable. The specific process is shown in Figure 1.

First, the algorithm is propagated forward. Calculate the output values of each neuron in the hidden layer and the output layer:

(1) $$\begin{array}{c} W_{j}=\underset{i}{\sum }w_{ji}u_{i}+b_{i}, \end{array}$$

(2) $$\begin{array}{c} u_{j}=f\left(W_{j}\right). \end{array}$$

Then, back propagation is carried out to calculate the error of each hidden layer neuron:

(3) $$\begin{array}{c} \delta_{j}=u_{j}\left(1-u_{j}\right)\underset{i}{\sum }w_{ij}\delta_{i}. \end{array}$$

*δ*_*j*_ is the sum of error information of all neurons in layer *j* + 1.

Finally, the weights of neurons are updated:

(4) $$\begin{array}{c} w_{ji}=w_{ji}-▲w_{ji}. \end{array}$$

#### 2.4.2. Support Vector Machine Model

In this study, the total hospitalization cost was a continuous variable, and the dependent variable should be discretized before the SVM fitting. The main parameters of the SVM model include penalty coefficient *C* and kernel function parameter *σ*. The selection of parameters in the SVM algorithm is very important to the learning performance of SVM. Reasonable parameter values can make SVM have higher training accuracy and stronger generalization ability. Therefore, this study will first screen out the optimal combination of *C* and *σ* parameters and establish the SVM model under the optimal combination of *C* and *σ* parameters. To select the optimal combination of *C* and *σ* parameters, the data is first normalized. Then, the data were input into the SVM model for verification to screen out the optimal combination. If the verification is inconsistent, the parameters need to be updated for verification again until the optimal combination is screened out. The SVM model building process is shown in Figure 2.

### 2.5. Statistical Analysis

One-way analysis was conducted on the relationship between the included research indicators and the total hospitalization expenses. Then, according to the results of the one-way analysis, significant variables are included in the BPNN model and SVM model as independent variables. After the training of the built models, the feature scores of associated predictors are screened out by machine learning.

## 3. Results

### 3.1. Analysis Results of Research Indicators

Univariate analysis was performed on the variables initially included. According to the results of medical payment method, hospitalization times, age, marital status, admission situation, critical illness during hospitalization, meet admission, and discharge, combined with other diagnosis, discharge departments, and receive surgical treatment have statistical significance (*P* < 0.05). Details are shown in Table 1.

However, gender, ethnicity, occupation, admission route, transfer department, complications, and discharge mode had no statistical significance on the total hospitalization cost (*P* > 0.05) (Table 2).

### 3.2. Results of Scoring Important Features in BPNN Algorithm Model

The results of BPNN model analysis show that the top three research indicators related to the total hospitalization expenses are hospitalization days (0.477), age (0.154), and discharge department (0.083). The characteristic scores of other research indicators are low (Figure 3).

### 3.3. Score Results of Important Features in SVM Algorithm Model

The results of the SVM algorithm model analysis show that the top three research indicators related to the total hospitalization expenses are hospitalization days (0.215), age (0.196), and marital status (0.172). The characteristic scores of other research indicators are low (Figure 4). As age may cause confounding of marital status, stratified analysis was conducted on age (≤25 years old and >25 years old) and marital status. The results showed that if age was controlled, the correlation between marital status and total hospitalization cost was not statistically significant (*P* > 0.05).

### 3.4. Distinction between BPNN Model and SVM Model

The area under the curve (AUC) of the BPNN model is 0.838 (95% CI: 0.755~0.921), which meets the prediction accuracy requirements. In comparison, the AUC of the SVM model is 0.889 (95% CI: 0.819~0.959) (Figure 5). The two prediction models have obtained a good prediction effect. However, the prediction efficiency of the SVM model is higher than the BPNN model.

## 4. Discussion

Bronchopneumonia is an infectious disease with a high incidence in China, especially among children. Its clinical manifestations are fever, cough, and shortness of breath, which affect the normal life [20]. It will not only affect the quality of life of patients but also bring a certain economic burden to families and pressure to the national medical insurance fund. Symptomatic treatment is a common intervention method with bronchopneumonia, which can effectively improve the symptoms and better control the development of the disease [21]. However, due to the younger age of patients, poor treatment compliance, and strong stress reaction, the hospitalization expenses are increased. Therefore, it is of specific clinical significance to predict the related indexes of total hospitalization expenses of patients with bronchopneumonia.

At present, the research on hospitalization expenses mainly includes traditional statistical methods, improved statistical methods, and machine learning methods [22, 23]. Traditional statistical methods have strict requirements on data, such as data normal and independent. Although nonparametric methods have no strict requirements on data characteristics, their efficiency is reduced because they do not use sample information to the maximum extent [24]. The improved statistical method combines other theories based on traditional methods and overcomes the inevitable defects of traditional methods to a certain extent. However, for some complex data, such as hierarchical data, subdepartment data, and doctor data within the hospital, the improved method is more complicated to calculate [25]. Before machine learning, we need to conduct a careful and in-depth preanalysis of the included data set. Otherwise, the results may be misleading. As a grey-box method, data mining can get correct results as long as researchers correctly master the input format of data and the way of reading the results, so it has perfect practicability [26].

In this study, the BPNN model and SVM model were used to analyze the total hospitalization cost of patients with bronchopneumonia, and good prediction results were obtained. The analysis of influencing factors pointed out that the length of stay and discharge department are two significant factors affecting the cost, which has practical guiding significance. The length of hospitalization is related to the severity of the disease and the effect of treatment, so it is necessary to improve the accuracy of treatment and rational use of antibacterial drugs in clinical practice. Different antibiotics can be selected for different patients at the beginning of admission according to their sputum culture results [27, 28]. For example, for older patients who have been exposed to antibiotics for a long time and higher-grade antibiotics can be selected to improve the treatment effect. For those with good physical quality and sensitivity to antibiotics, low-grade antibiotics can be selected appropriately [29]. The different treatment methods and medication habits of doctors in different departments lead to the difference in total hospitalization expenses [30]. Therefore, it is recommended that doctors select appropriate treatment plans for patients. At the same time, the patient's age is also a major factor affecting hospitalization expenses. This is mainly because older patients have more comorbidities, relatively poor resistance, and low sensitivity to drugs, so there are relatively more drugs in the treatment process, resulting in prolonged hospitalization days and increased hospitalization expenses [31]. The results of the SVM model in this study showed that marital status was a major factor affecting the total hospitalization cost. Still, there was no statistical significance after stratified analysis and control of confounding factors.

The AUC of the prediction models was also compared in our study. The results show that the AUC of these two models is 0.838 (95% CI: 0.755~0.921) and 0.889 (95% CI: 0.819~0.959), respectively. It further shows that the prediction effect of SVM is better than the BPNN model. The reason may be that the SVM pursues optimal solutions under existing information and can perfectly solve high and local extremum problems [32]. The SVM overcomes the defects of the BPNN method, such as the difficulty in determining the reasonable structure and the existence of local optimum, especially for the data with dependent variables as classification variables, and has been effectively used in practice [17].

There are several limitations to our study. First, the specimens included were too small and from the same region. In addition, the incompleteness of the included predictors may directly affect the prediction results after deep learning. In future research, the sample size and prediction factors will be increased.

## 5. Conclusion

In conclusion, BPNN and SVM prediction models can effectively predict the total cost of hospitalized patients, and the most critical factor affecting the total cost of hospitalization is the length of stay. Therefore, shortening the length of stay may minimize the financial burden of patients.

## Figures and Tables

**Figure 1:** BP neural network construction flow chart.

**Figure 2:** SVM model training process chart.

**Figure 3:** Score of important features in BPNN algorithm model.

**Figure 4:** Score of important features in SVM algorithm model.

**Figure 5:** ROC curve of BPNN model and SVM model.

**Table 1:** Analysis results related to total hospitalization expenses of patients with bronchopneumonia.

Research indicators	*χ* ^2^/*F*	*P*
Medical payment method	151.359	0.023
Hospitalization times	0.652	0.038
Age	0.166	<0.001
Marital status	-18.791	<0.001
Admission situation	35.515	0.036
Critical illness during hospitalization	-11.746	0.027
Meet admission and discharge	-4.290	0.041
Combined with other diagnoses	-12.210	0.026
Discharge departments	421.631	0.048
Receive surgical treatment	-4.256	0.015

**Table 2:** Analysis results unrelated to the total hospitalization expenses of patients with bronchopneumonia.

Research indicators	*χ* ^2^/*F*	*P*
Gender	-0.314	0.814
Ethnicity	-0.325	0.792
Occupation	3.540	0.357
Admission route	3.451	0.069
Transfer department	4.259	0.071
Complications	-2.452	0.216
Discharge mode	2.421	0.255

## Data Availability

The data used to support the findings of this study are available from the corresponding author upon request.

## References

[1] Rutenberg D., Venner M., Giguère S. (2017). Efficacy of tulathromycin for the treatment of foals with mild to moderate bronchopneumonia. *Journal of Veterinary Internal Medicine*.

[2] Wang Y., Sun Y., Zhang H., Yang X., Song X. (2021). Comprehensive analysis of the diagnosis and treatment of tracheobronchial foreign bodies in children. *Ear, Nose, & Throat Journal*.

[3] You C., Ran G., Wu X. (2019). High immunoglobulin e level is associated with increased readmission in children with bronchopneumonia. *Therapeutic Advances in Respiratory Disease*.

[4] Han X., Yang Y., Zhu Q., Wang X., Huang W. (2022). Clinical value of atomization therapy in children with bronchopneumonia. *Minerva Pediatr (Torino)*.

[5] Lindström L., Tauni F. A., Vargmar K. (2018). Bronchopneumonia in Swedish lambs: a study of pathological changes and bacteriological agents. *Acta Veterinaria Scandinavica*.

[6] Ye J., Ye H., Wang M., Zhao Y. (2021). Total serum il-6 and tnf-c levels in children with bronchopneumonia following treatment with methylprednisolone in combination with azithromycin. *American Journal of Translational Research*.

[7] Aziz D. A., Billoo A. G., Qureshi A., Khalid M., Kirmani S. (2017). Clinical and laboratory profile of children with cystic fibrosis: experience of a tertiary care center in Pakistan. *Pak J Med Sci*.

[8] Shen Z., Zhang Y., Li H., Du L. (2022). Rapid typing diagnosis and clinical analysis of subtypes a and b of human respiratory syncytial virus in children. *Virology Journal*.

[9] Buja A., Bardin A., Grotto G. (2021). How different combinations of comorbidities affect healthcare use by elderly patients with obstructive lung disease. *NPJ Prim Care Respir Med*.

[10] Chen K. C., Yu H. R., Chen W. S. (2020). Diagnosis of common pulmonary diseases in children by X-ray images and deep learning. *Scientific Reports*.

[11] Schalekamp S., Klein W. M., van Leeuwen K. G. (2021). Current and emerging artificial intelligence applications in chest imaging: a pediatric perspective. *Pediatric Radiology*.

[12] Ye Y., Shi J., Zhu D., Su L., Huang J., Huang Y. (2021). Management of medical and health big data based on integrated learning-based health care system: a review and comparative analysis. *Computer Methods and Programs in Biomedicine*.

[13] Wang D., Fong S., Wong R. K., Mohammed S., Fiaidhi J., Wong K. K. (2017). Robust high-dimensional bioinformatics data streams mining by odr-iovfdt. *Scientific Reports*.

[14] Chuang L. Y., Yang C. H., Tsai J. H., Yang C. H. (2013). Operon prediction using chaos embedded particle swarm optimization. *IEEE/ACM Transactions on Computational Biology and Bioinformatics*.

[15] Zhao D., Chen M., Shi K., Ma M., Huang Y., Shen J. (2021). A long short-term memory-fully connected (lstm-fc) neural network for predicting the incidence of bronchopneumonia in children. *Environmental Science and Pollution Research International*.

[16] Nedaie A., Najafi A. A. (2018). Support vector machine with Dirichlet feature mapping. *Neural Networks*.

[17] Bao C., Pu Y., Zhang Y. (2018). Fractional-order deep backpropagation neural network. *Comput Intell Neurosci*.

[18] Gong E., Pauly J. M., Wintermark M., Zaharchuk G. (2018). Deep learning enables reduced gadolinium dose for contrast-enhanced brain MRI. *Journal of Magnetic Resonance Imaging*.

[19] Tian S. K., Dai N., Li L. L., Li W. W., Sun Y. C., Cheng X. S. (2020). Three-dimensional mandibular motion trajectory-tracking system based on bp neural network. *Mathematical Biosciences and Engineering*.

[20] Jeong J. E., Soh J. E., Kwak J. H. (2018). Increased procalcitonin level is a risk factor for prolonged fever in children with mycoplasma pneumonia. *Korean Journal of Pediatrics*.

[21] Liu X., Meng J. (2018). Luteolin alleviates LPS-induced bronchopneumonia injury _in vitro_ and _in vivo_ by down-regulating microRNA-132 expression. *Biomedicine & Pharmacotherapy*.

[22] Lee S., Lim H. (2019). Review of statistical methods for survival analysis using genomic data. *Genomics Inform*.

[23] Zhou Z. R., Wang W. W., Li Y. (2019). In-depth mining of clinical data: the construction of clinical prediction model with r. *Ann Transl Med*.

[24] Grendas L. N., Chiapella L., Rodante D. E., Daray F. M. (2021). Comparison of traditional model-based statistical methods with machine learning for the prediction of suicide behaviour. *Journal of Psychiatric Research*.

[25] Qiu X., Gao J., Yang J., Hu J., Hu W., Kong L. (2020). A comparison study of machine learning (random survival forest) and classic statistic (cox proportional hazards) for predicting progression in high-grade glioma after proton and carbon ion radiotherapy. *Frontiers in Oncology*.

[26] Verma A. K., Pal S., Kumar S. (2020). Prediction of skin disease using ensemble data mining techniques and feature selection method-a comparative study. *Applied Biochemistry and Biotechnology*.

[27] Rolsma S. L., Rankin D. A., Haddadin Z. (2021). Assessing the epidemiology and seasonality of influenza among children under two hospitalized in Amman, Jordan, 2010-2013. *Influenza and Other Respiratory Viruses*.

[28] Zhang L., Lai M., Ai T. (2021). Analysis of mycoplasma pneumoniae infection among children with respiratory tract infections in hospital in Chengdu from 2014 to 2020. *Transl Pediatr*.

[29] Kudagammana S. T., Karunaratne R. R., Munasinghe T. S., Kudagammana H. (2020). Community acquired paediatric pneumonia; experience from a pneumococcal vaccine- naive population. *Pneumonia (Nathan)*.

[30] Wetzig M., Venner M., Giguère S. (2020). Efficacy of the combination of doxycycline and azithromycin for the treatment of foals with mild to moderate bronchopneumonia. *Equine Veterinary Journal*.

[31] Lu Y., Wang Y., Hao C. (2018). Clinical characteristics of pneumonia caused by mycoplasma pneumoniae in children of different ages. *International Journal of Clinical and Experimental Pathology*.

[32] Huang S., Cai N., Pacheco P. P., Narrandes S., Wang Y., Xu W. (2018). Applications of support vector machine (svm) learning in cancer genomics. *Cancer Genomics Proteomics*.

